RETRACTED

# Metformin-Enhanced Cardiac AMP-Activated Protein Kinase/Atrogin-1 Pathways Inhibit Charged Multivesicular Body Protein 2B Accumulation in Ischemia–Reperfusion Injury

**DOI:** 10.3389/fcell.2020.621509

**Published:** 2021-02-05

**Authors:** Tian Li, Yue Yin, Nan Mu, Yishi Wang, Manling Liu, Mai Chen, Wenhua Jiang, Lu Yu, Yan Li, Heng Ma

**Affiliations:** ^1^Department of Physiology and Pathophysiology, Fourth Military Medical University, Xi'an, China; ^2^Department of Cardiovascular Medicine, Xijing Hospital, Fourth Military Medical University, Xi'an, China; ^3^Institute of Medical Research, Northwestern Polytechnical University, Xi'an, China; ^4^Department of Pathology, Xijing Hospital, Fourth Military Medical University, Xi'an, China; ^5^Department of Cardiovascular Medicine, Tangdu Hospital, Fourth Military Medical University, Xi'an, China

**Keywords:** myocardial ischemia/reperfusion, metformin, autophagic flux, AMPK, atrogin-1, CHMP2B

## Abstract

**Background:** Cardiac autophagic flux is impaired during myocardial ischemia/reperfusion (MI/R). Impaired autophagic flux may exacerbate MI/R injury. Charged multivesicular body protein 2B (CHMP2B) is a subunit of the endosomal sorting complex required for transport (ESCRT-III) complex that is required for autophagy. However, the reverse role of CHMP2B accumulation in autophagy and MI/R injury has not been established. The objective of this article is to elucidate the roles of AMP-activated protein kinase (AMPK)/atrogin-1 pathways in inhibiting CHMP2B accumulation in ischemia–reperfusion injury.

**Methods:** Male C57BL/6 mice (3–4 months) and H9c2 cardiomyocytes were used to evaluate MI/R and hypoxia/reoxygenation (H/R) injury *in vivo* and *in vitro*, respectively. MI/R was built by a left lateral thoracotomy and occluded the left anterior descending artery. H9c2 cells were firstly treated in 95% N_2_ and 5% CO_2_ for 15 h and reoxygenation for 1 h. Metformin (100 mg/kg/d) and CHMP2B (Ad-CHMP2B) transfected adenoviruses were administered to the mice. The H9c2 cells were treated with metformin (2.5 mM), MG-132 (10 μM), bafilomycin A1 (10 nM), and compound C (20 μM).

**Results:** Autophagic flux was found to be inhibited in H/R-treated cardiomyocytes and MI/R mice, with elevated cardiac CHMP2B accumulation. Upregulated CHMP2B levels in the *in vivo* and *in vitro* experiments were shown to inhibit autophagic flux leading to the deterioration of H/R-cardiomyocytes and MI/R injury. This finding implies that CHMP2B accumulation increases the risk of myocardial ischemia. Metformin suppressed CHMP2B accumulation and ameliorated H/R-induced autophagic dysfunction by activating AMPK. Activated AMPK upregulated the messenger RNA expression and protein levels of atrogin-1, a muscle-specific ubiquitin ligase, in the myocardium. Atrogin-1 significantly enhanced the interaction between atrogin-1 and CHMP2B, therefore, promoting CHMP2B degradation in the MI/R myocardium. Finally, this study revealed that metformin-inhibited CHMP2B accumulation induced autophagic impairment and ischemic susceptibility *in vivo* through the AMPK-regulated CHMP2B degradation by atrogin-1.

RETRACTED

**Conclusion:** Impaired CHMP2B clearance *in vitro* and *in vivo* inhibits autophagic flux and weakens the myocardial ischemic tolerance. Metformin treatment degrades CHMP2B through the AMPK-atrogin-1-dependent pathway to maintain the homeostasis of autophagic flux. This is a novel mechanism that enriches the understanding of cardioprotection.

## Introduction

Globally, ischemic heart disease is among the leading causes of mortality and disability (Collaborators, 2018). Ischemic injury-induced cardiomyocyte death leads to a permanent loss of the cardiac functional unit and, ultimately, heart failure (Del Re et al., 2019). Cardiomyocytes are terminally differentiated cells that fail to regenerate through mitosis. Abnormal events-associated protein instability leads to efficient and accurate protein degradation/reuse, which is necessary for cardiomyocytes to maintain physiological functions (Li C. et al., 2020).

The ubiquitin–proteasome system (UPS) and autophagy are two major cell quality control pathways. Parallel to the UPS, autophagy is a lysosome-dependent bulk degradation system that inhibits the abnormal accumulation of intracellular proteins and organelles. It is an important process for cellular self-renewal, dynamic energy equilibrium, the maintenance of functional homeostasis, and cardiomyocyte survival (Chang, 2020; Oeing et al., 2020). Autophagic flux loss-of-function enhances cardiac dysfunction that is accompanied by the accumulation of misfolded proteins and dysfunctional organelles (Shirakabe et al., 2016). Our previous studies established that impaired autophagic flux sensitizes the heart to myocardial ischemia/reperfusion (MI/R) injury. MI/R injury can also disrupt autophagic functions (Wang et al., 2019; Li C. et al., 2020). Therefore, actively improving functional cardiac autophagy during MI/R is an effective myocardial protection strategy.

The endosomal sorting complex required for transport (ESCRT) protein complexes have been reported to exhibit an effect on lysosome–autophagosome fusion (Zaglia et al., 2014). Charged multivesicular body protein 2B (CHMP2B) is a subunit of ESCRT-III that mediates proteasome degradation and autophagy (Wiersma et al., 2019; Feng et al., 2020). Ectopic expression of CHMP2B disrupts autophagy and is associated with frontotemporal dementia (Lee and Gao, 2009), whereas dominant mutations in CHMP2B (CHMP2BIntron5) are associated with a subset of heritable frontotemporal dementia (Krasniak and Ahmad, 2016). However, the roles of CHMP2B in the myocardium have not been elucidated. Previous studies revealed the roles of CHMP2B in the formation of autophagic vesicles. It is important to establish what happens to the cell when CHMP2B accumulates due to inhibited autophagy.

RETRACTED

Metformin is a first-line antidiabetic drug with pro-autophagic and cardioprotective effects. Metformin protects against MI/R injury by activating AMP protein kinase (AMPK) (Wang et al., 2019; Li C. et al., 2020). The protective effects of AMPK on the cardiovascular system have been reviewed (Li et al., 2017; Gu et al., 2018; Jiang et al., 2018; Li T. et al., 2020). Also, we confirmed that metformin enhances autophagic function in the aging myocardium (Li C. et al., 2020). However, it is not clear whether metformin maintains the homeostasis of myocardial autophagy during MI/R by regulating CHMP2B. Therefore, this study aimed at: (i) determining the association between myocardial CHMP2B levels, myocardial autophagy function, and myocardial injury during MI/R; (ii) establishing whether the accumulation of CHMP2B impairs myocardial autophagy and aggravates MI/R injury; and (iii) evaluating whether metformin protects against MI/R injury by regulating CHMP2B and autophagic flux.

## Materials and Methods

### Animals and Human Data

Male C57BL/6J mice (3–4 months old) were purchased from the Experimental Animal Center of the Fourth Military Medical University. Ethical approval for the use of animals in this study was obtained from the Animal Ethical Experimentation Committee of the Fourth Military Medical University (IACUC-20200602). Animals were housed under a 12:12-h light/dark cycle with *ad libitum* access to a regular pellet diet. The mice were randomly assigned to each experimental group. Using normal saline as the vehicle, metformin hydrochloride (Solarbiol, Beijing, China, 100 mg/kg/day) was intraperitoneally administered to the mice daily, for 7 days as previously described (Chen et al., 2017). The control mice were administered with saline.

Human data were obtained from the Open Access database of National Center for Biotechnology Information. Total RNA samples obtained from the peripheral blood of coronary heart disease (CAD) patients and healthy controls among the Chinese Han people and deposited in Gene Expression Omnibus (GEO) were assessed through the GEO Series accession number GSE71226. We reanalyzed these data using a volcano plot.

RETRACTED

### *In vivo* Ischemia and Reperfusion Surgery

MI/R mice model was established as previously described (Li C. et al., 2020). Mice were anesthetized with 2% isoflurane, intubated, and ventilated using a rodent ventilator (Taimeng Co., Ltd., Chengdu, China). A left lateral thoracotomy was performed and the left anterior descending artery occluded using a 7–0 nylon suture for 30 min of ischemia, followed by 2 h (signaling evaluation) or 4 h (morphological analysis) after reperfusion.

### Cell Culture and Hypoxia/Reoxygenation

H9c2 cells (Cell Bank, Chinese Academy of Sciences, Shanghai, China), a subclone of the original clonal cell line derived from embryonic BD1X rat heart tissue, were cultured in Dulbecco's modified Eagle's medium (Gibco) that had been supplemented with 10% fetal bovine serum (Gibco) and 1% penicillin–streptomycin mixture (Solarbiol, Beijing, China). The cell culture was incubated in a 5% CO_2_ atmosphere at 37°C. The growth medium was changed every 2 days, and the cells were experimentally used once they reached a 70–80% confluence. They were incubated with the vehicle, metformin (2.5 mM) (Salani et al., 2017), and compound C (20 μM) for 12 h (Hao et al., 2019). For hypoxia/reoxygenation (H/R) treatment, the H9c2 cells were first treated in 95% N_2_ and 5% CO_2_ (Modular Incubator Chamber, Billups-Rothenberg, Inc., Del Mar, CA, USA) for 15 h and reoxygenated (95% air and 5% CO_2_) for 1 h (Chen et al., 2018).

### Western Blotting and Immunoprecipitation

Rabbit p-AMPKα (#2535), AMPKα (#5832), CHMP2B (#76173), α-tubulin (#9099), p62 (#16177), LC3B (#3868), and Atg 5 (#12994) antibodies were purchased from Cell Signaling Technology (Danvers, MA, USA); rabbit atrogin-1 (Muscle atrophy box F gene 1, ab168372) and LAMP1 (ab24170) antibodies were purchased from Abcam (Cambridge, MA, USA); sheep anti-CHMP2B (AF7509) for immunofluorescence was purchased from R&D System (Minneapolis, MN, USA), whereas all primary MG-132 (10 μM) (Xu et al., 2016) and bafilomycin A1 (Baf-A1, 10 nM) (Wong et al., 2019) were purchased from MCE (Monmouth Junction, NJ, USA). Western blotting was performed as previously described (Chang et al., 2019). Immunoprecipitation was performed using an Immunoprecipitation Kit-Dynabeads Protein G according to the manufacturer's protocol (Invitrogen, Carlsbad, CA, USA). The enhanced chemiluminescence detection kit was obtained from Millipore (Darmstadt, Germany).

### Immunohistochemistry and Immunofluorescence

Immunofluorescence staining, immunohistochemistry of cardiac sections, and H9c2 cell immunofluorescence were performed as previously described (Yan et al., 2017; Zhao et al., 2020).

### Cell Viability

The CCK-8 (Solarbiol, Beijing, China) assay was performed to quantitatively evaluate cell viability as previously described (Chang et al., 2019). Briefly, 100-μl medium of H9c2 cells was replaced with fresh culture medium. Ten microliters of CCK-8 solution was then added into each well. After incubation for 1 h at 37°C, absorbance at 450 nm was determined using a microplate reader (Molecular Devices, CA, USA).

RETRACTED

### Assay of Cardiac Injury

Blood samples for CK-MB activity and lactate dehydrogenase (LDH) concentrations were collected 24 h after MI/R and analyzed spectrophotometrically as previously described (Gu et al., 2013; Xing et al., 2016).

### Adenovirus Delivery

H9c2 cells were transfected with adenovirus-expressing CHMP2B (Ad-CHMP2B) (GemmaPharma, Shanghai, China) as previously described (Shimizu et al., 2016). The adenovirus titers used in this study were 1.0 × 10^10^ PFU/ml, whereas the multiplicity of infection was 100:1. Forty-eight hours after transfection, the cells were subjected to experimental administration of metformin.

Rattus Flag-CHMP2B plasmid and Myc-Atrogin1 plasmid (RR212771, OriGene, Rockville, MD, USA) were used for immunoprecipitation purposes. The complete open reading frame of rattus CHMP2B was constructed by DNA synthesis containing Not I and Kpn I restriction sites within the 5′ and 3′ termini (Sangon, Shanghai, China). Synthetic complementary DNA was inserted into the pFlag-CMV-2 vector. A green fluorescent protein (GFP)-mRFP-LC3 virus is an adenovirus tool for researching autophagy flux (20812860). Cells were treated with GFP-mRFP-LC3 adenovirus (1.0 × 1,010 PFU/ml, HanBiol, Shanghai, China) with a multiplicity of infection as 100:1. Forty-eight hours after transfection, the cells were subjected to experimental administration of metformin (Control, H/R + V, H/R + M), as previously described. When mRFP-GFP-LC3 fusion proteins fuse with acidic lysosomes, red fluorescence is observed, and GFP is quenched. A yellow fluorescence is observed when autophagosomal clearance is impaired.

### Flow Cytometry Assay

Cells were collected by tyrisin (Solarbiol, Beijing, China), washed thrice using phosphate-buffered saline, stained using the AnnexinV-FITC/PI apoptosis detection kit (BD Biosciences, San Jose, CA, USA) and analyzed in a FACSCalibur flow cytometer (BD Biosciences, San Jose, CA, USA).

### Quantitative Real-Time PCR

RNA extraction and real-time quantitative PCR were performed as previously described (Yan et al., 2013). The primer sequences used in this study were as follows (5′−3′): atrogin-1 forward GGGAGTACTAAGGAGCGCCA, reverse TCTGGACCAGCGTGCATAAG; actin forward GTCCCTCACCCTCCCAAAAG, reverse GCTGCCTCAACACCTCAACCC.

RETRACTED

### Echocardiography and Electrocardiography

Echocardiography was performed using Vevo 2100 (Visual Sonics, Toronto, ON, Canada) as previously described (Ding et al., 2017). Mice were anesthetized using 2% isoflurane. *In vivo* transthoracic echocardiography of the left ventricle was used to obtain high-resolution two-dimensional mode images. Left ventricular fractional shortening and ejection fraction in M-mode images were measured.

### Statistical Analysis

All data were presented as mean ± standard error of the mean. One-way analysis of variance, followed by Dunnett's test *post-hoc* test, was used to determine statistical differences among groups. All statistical analyses were performed using GraphPad Prism 8.0 (GraphPad Software, San Diego, CA, USA). A *p* ≤ 0.05 was considered to be statistically significant.

## Results

### Metformin Prevents Hypoxia/Reoxygenation-Induced Cardiomyocyte Autophagy Flux Inhibition and Cellular Injury

The accumulation of autophagosomes has been reported to promote cardiomyocyte death. To evaluate autophagic flux impairment due to H/R-induced injury in cardiomyocytes, the *in vitro* state of the autophagy/lysosomal system under H/R condition was evaluated. We found that the expression levels of Atg 5, LC3 II/I, LAMP1, and p62 were significantly elevated in H/R-treated H9c2 cells (Figure 1A), suggesting that autophagic flux was impaired. Autophagosome accumulation was confirmed by the fluorescence results (Figure 1B, Supplementary Figure 1). Treatment with metformin was found to inhibit autophagic flux impairment. Metformin (2.5 mM) (Salani et al., 2017) was administered to H9c2 cells for 16 h. The cells were concurrently subjected to H/R injury. Compared with the H/R group, metformin treatment markedly decreased H/R cardiomyocyte p62 levels associated with low Atg5, LC3 II/I, and LAMP2 levels as well as decreased GFP-RFP-LC3 (yellow fluorescence) (Figures 1A,B and Supplementary Figure 1). Furthermore, metformin treatment protected against H/R-induced cardiomyocyte injury increased cell viability and suppressed CK-MB activity as well as LDH concentration levels (Figure 1C).

**Figure 1:** Metformin prevents H/R-induced cardiomyocyte autophagic flux blocking and injury. H9c2 cells were treated with metformin (2.5 mmol/L) or vehicle for 12 h and subjected to hypoxia for 15 h followed by reoxygenation for 1 h. **(A)** Representative Western blot and quantification data for Atg 5, LC3 II/I, LAMP1, and p62 in H9c2 cells; tubulin was used as loading control. **(B)** Representative images of fluorescent LC3 puncta after mRFP-GFP-LC3 adenovirus transduction (24 h) and analysis of the autophagosome and autophagolysosome in control cells or subjected to H/R with or without metformin treatment. **(C)** Quantification data for cell viability, CK-MB activity, and LDH concentration were calculated for control cells or cells subjected to H/R with or without metformin treatment. M, metformin; V, vehicle; H/R, hypoxia/reoxygenation; RLU, relative light unit; GFP, green fluorescent protein; RFP, red fluorescent protein; DAPI, 2-(4-Amidinophenyl)-6-indolecarbamidine dihydrochloride. Scale bar = 10 μm. Values are means ± SEM, *n* = 6 per group, *p ≤ 0.05 vs. control group, ^#^*p* ≤ 0.05 vs. tH/R + vehicle group.

RETRACTED

### Charged Multivesicular Body Protein 2B Accumulated in Hypoxia/Reoxygenation-Treated Cardiomyocytes and Was Upregulated in Coronary Heart Disease Patients

Compared with the control, CHMP2B levels were found to be significantly elevated (3.8-fold) in H/R-induced autophagy-impaired cardiomyocytes (Figure 2A). Metformin treatment suppressed CHMP2B levels and restored autophagy in H/R-treated cardiomyocytes (Figure 2A).

**Figure 2:** CHMP2B accumulated in hypoxia/reoxygenation and in patients with coronary heart disease. **(A)** Representative immunoblotting and quantification data of CHMP2B levels in control cells and those subjected to H/R with or without metformin treatment. **(B)** Total RNA samples from three CAD patients and three healthy people of the Chinese Han population were extracted from peripheral blood and hybridized with Affymetrix microarrays. Volcano plot shows that mRNA expression levels of CHMP2B were upregulated in CAD patients, ~1.9-fold. **(C)** Fold change of CHMP2B mRNA from three CAD patients and three healthy people. We reanalyzed data from GEO database (GSE71226) for two microarray sites. Values are the means ± SEM, *n* = 6 per group, *p ≤ 0.05 vs. control group, ^#^*p* ≤ 0.05 vs. H/R + vehicle group.

Moreover, we reanalyzed clinical data from CAD patients (Zeng et al., 2013). The microarray results revealed upregulated CHMP2B RNA levels in CAD patients. This upregulation was ~1.9-fold than in healthy people (Figures 2B,C). Therefore, these results imply that CHMP2B accumulation is associated with autophagic dysfunction and ischemic injury.

### Charged Multivesicular Body Protein 2B Overexpression Impairs Autophagic Flux in Cardiomyocytes, Leading to Myocardial Vulnerability to Ischemia/Reperfusion

We evaluated the functional relationship between autophagic inhibition and CHMP2B accumulation. H9c2 cells were infected with control adenovirus (Ad-Con) or Ad-CHMP2B for 48 h. Adenovirus-infected cells are GFP-positive (Supplementary Figure 2). Adenovirus-mediated overexpression of CHMP2B markedly elevated the protein levels of LC3 II/I, LAMP1, and p62 in cells (Figure 3A). Autophagic flux was assessed by treatment with Baf-A1. Baf-A1 treatment (48 h) increased LC3 II/I and p62 protein levels in the Ad-Con group. However, it did not exhibit any significant changes on CHMP2B overexpressed cardiomyocytes (Figure 3B), implying that excessive CHMP2B disrupts autophagic flux. CHMP2B-associated autophagic flux inhibition enhanced H/R-induced myocardial cell death (Figure 3C). These results reveal that although CHMP2B mediates autophagy under basal conditions, excess CHMP2B accumulation inhibits autophagic flux and enhances H/R-induced cardiomyocyte death.

RETRACTED

**Figure 3:** Overexpressed CHMP2B impairs autophagic flux leading to myocardial susceptibility to ischemia. H9c2 cells were infected with control adenovirus (Ad-Con) or CHMP2B-transfected adenovirus (Ad-CHMP2B) for 48 h. **(A)** Representative immunoblotting and quantification data of CHMP2B, LC3 II/I, LAMP1, and p62 were compared with normal control, Ad-Control, or Ad-CHMP2B treatment. **(B)** Ad-Con or Ad-CHMP2B cardiomyocytes were subjected to bafilomycin A1 (10 nM) or DMSO vehicle treatment. Representative immunoblotting and quantification data of CHMP2B, LC3 II/I, and p62. **(C)** Cell death rate was determined by annexin V-FITC/PI staining assay. B2 + B4 means apoptotic cells. Representative images obtained by flow cytometric analysis are shown on left side. Statistical analysis of percentage of apoptotic cells in different groups is shown on the right. Values are the means ± SEM, *n* = 6 per group. Except as otherwise noted, *p ≤ 0.05 vs. control or Ad-Con group, ^#^*p* ≤ 0.05 vs. control + HR or Ad-Con + HR group. BAf-A1, Bafilomycin A1; DMSO, dimethylsulfoxide.

### Metformin Prevented Charged Multivesicular Body Protein 2B Accumulation in Hypoxia/Reoxygenation-Treated Cardiomyocytes Through the AMP-Activated Protein Kinase Pathway

Metformin treatment significantly enhanced the phosphorylation of AMPK in H/R-treated cardiomyocytes, enhanced the expression of atrogin-1 (a muscle-specific ubiquitin ligase) (Elsaid et al., 2017; Li C. et al., 2020), and suppressed the accumulation of CHMP2B in H/R cardiomyocytes (Figure 4A). Furthermore, through the AMPK pathway, metformin upregulated atrogin-1 protein and messenger RNA (mRNA) expression levels (Figures 4B,C) while suppressing CHMP2B levels. However, these effects were blocked by the AMPK activity blocker compound C (20 μM) (Figures 4B,C). AMPK inhibitor resulted in decreased autophagic induction and degradation of cardiomyocytes, which was consistent with the feature of autophagy flux blocking (Supplementary Figure 3). We also found that atrogin-1 and CHMP2B were co-localized in cardiomyocytes. Fluorescent co-localization of atrogin-1 and CHMP2B was significantly enhanced by metformin treatment during H/R injury (Figure 4D). These findings indicate that atrogin-1 directly interacts with CHMP2B, and metformin regulates this process by activating AMPK under H/R condition.

RETRACTED

**Figure 4:** Metformin prevents CHMP2B accumulation in H/R-treated cardiomyocytes in AMPK dependent manner. H9c2 cells were treated with metformin (2.5 mmol/L) or vehicle for 12 h and subjected to hypoxia for 15 h followed by reoxygenation for 1 h. **(A)** Representative immunoblotting and quantification data of p-AMPKα, AMPKα, atrogin-1, and CHMP2B for each group. **(B)** H9c2 cells were treated with metformin (2.5 mmol/L) or compound C (20 μmol/L) for 12 h. Representative immunoblotting and quantification data of p-AMPKα, AMPKα, atrogin-1, and CHMP2B for each group. **(C)** Relative mRNA expression levels of atrogin-1 as determined by qRT-PCR. **(D)** H9c2 cells were treated with metformin (2.5 mmol/L) or vehicle and simultaneously subjected to hypoxia for 15 h followed by reoxygenation for 1 h. Representative photomicrographs for CHMP2B (green) and atrogin-1 (red) co-localization staining by immunofluorescence. Scale bar = 50 μM. Values are means ± SEM, *n* = 6 per group. Except as otherwise noted, *p ≤ 0.05 vs. control group, ^#^*p* ≤ 0.05 vs. H/R + vehicle or compound C group.

### Charged Multivesicular Body Protein 2B Is Degraded by Atrogin-1

We confirmed the interaction between atrogin-1 and CHMP2B through *in vitro* experiments. Flag-tagged CHMP2B coimmunoprecipitated with Myc-tagged atrogin-1 in atrogin-1 and CHMP2B co-transfected cells (Figure 5A). Cardiomyocytes were treated with the proteasome inhibitor MG-132 (10 μM), which caused CHMP2B polyubiquitination (Figure 5B) and time-dependent accumulation (Figure 5D). Our *in vivo* experiments confirmed the interaction between atrogin-1 and CHMP2B (Figures 5C,E). These results support the concept that CHMP2B is a ubiquitination degradation target for atrogin-1 in the cardiomyocytes.

**Figure 5:** Binding relationship exists between atrogin-1 and CHMP2B. **(A)** Immunoprecipitation was performed to evaluate the relationship between atrogin-1 and CHMP2B. H9c2 cells transfected with Myc-atrogin-1 and Flag-CHMP2B were subjected to immunoblotting analysis. **(B)** H9c2 cells were treated with MG-132 for 24 h (10 μM) and harvested for immunoprecipitation purposes using ubiquitin primary antibody. **(C)** H9c2 cells were treated with MG-132 (10 μM) for 12 or 24 h and representative immunoblots of CHMP2B and ubiquitin obtained. **(D)** Quantification data of CHMP2B and ubiquitin in pattern **(C)**. **(E)** Representative co-immunoprecipitation analysis of CHMP2B and atrogin-1 in cardiacs from C57 mice. Mixture of bead and CHMP2B primary antibody were acquired and incubated with atrogin-1 primary antibody overnight. Arrow shows molecular weight of 42 kD (atrogin-1). Values are means ± SEM, *n* = 6 per group. Except as otherwise noted, *p ≤ 0.05 vs. control group. IgH, immunoglobulin heavy chain; IgL, immunoglobulin light chain.

RETRACTED

### *In vivo* Charged Multivesicular Body Protein 2B Accumulation Impairs Autophagic Flux and Worsens Myocardial Ischemia/Reperfusion Injury

Three-month-old C57 WT mice were ventricularly administered with an Ad-CHMP2B or Ad-Con for 48 h and GFP to label the infected myocardial tissues. The immunofluorescence and immunohistochemistry results revealed that the overexpression *in vivo* model of Ad-CHMP2B was successfully established (Figures 6A,B). It was found that overexpressed CHMP2B did not exert any effect on AMPK phosphorylation or atrogin-1 expression. However, LC3 II/I and p62 levels in the myocardial tissue were significantly elevated and were maintained at an elevated level during MI/R (Figure 6C). In the *in vivo* experiments, overexpressed CHMP2B was found to significantly aggravate MI/R injury, as shown by the low myocardial contraction and relaxation (indicated by decreased ejection fraction and fractional shortening, Figure 6D), high LDH secretion (Figure 6E), and CK-MB levels (Figure 6F), as well as the serious arrhythmia indices (Figure 6G). Overexpressed CHMP2B significantly elevated the mortality rate in MI/R injured mice (Figure 6H). We also found that overexpression of CHMP2B impairs autophagic flux, and the cardioprotective effect of metformin can be counteracted by CHMP2B overexpression under MI/R and H/R (Supplementary Figures 5, 6).

**Figure 6:** CHMP2B accumulation impairs autophagic flux and worsens myocardial MI/R injury *in vivo*. C57 mice were ventricularly injected with an adenovirus vector encoding CHMP2B (Ad-CHMP2B) or Ad-Con as a control. **(A)** Adenovirus-infected hearts exhibited GFP-positive myocardium, Scale bar: 50 μM. **(B)** Immunochemistry results showed that CHMP2B was successfully overexpressed 72 h after Ad-CHMP2B rejection. Scale bar: 100 μM. **(C)** C57 mice were intramyocardially injected with Ad-CHMP2B or Ad-Con 72 h before MI/R surgery (ischemia for 30 min and reperfusion for 120 min). Representative immunoblots and quantification data of p-AMPKαM AMPKα, atrogin-1, CHMP2B, p62, and LC3 II/I. **(D)** Representative photomicrographs and average data for left ventricle ejection fraction (LVEF) and fractional shortening (LVFS) were assessed by echocardiography in Ad-CHMP2B- or Ad-Con-injected mice subjected to sham or MI/R injury (30 min of ischemia and 4 weeks of reperfusion). **(E)** LDH concentrations, **(F)** CK-MB activity, **(G)** arrhythmia index for each group (ischemia 30 min and reperfusion 240 min). **(H)** Survival curve for Ad-Con, Ad-CHMP2B, MI/R + Ad-Con, and MI/R + Ad-CHMP2B groups (*p* < 0.05). Values are means ± SEM, *n* = 6–9 per group. Except as otherwise noted, *p ≤ 0.05 vs. sham + Ad-Con group. ^#^*p* ≤ 0.05 vs. MI/R + Ad-Con group.

RETRACTED

### Metformin-Enhancing Cardiac AMP-Activated Protein Kinase/Atrogin-1 Pathways Prevent Charged Multivesicular Body Protein 2B Accumulation in Myocardial Ischemia/Reperfusion Injury

The results described earlier suggest that CHMPB accumulation inhibits autophagy and aggravates MI/R injury. Therefore, we aimed to establish whether metformin can prevent accumulated CHMPB-associated autophagy and enhance myocardial resistance to MI/R damage. Metformin (100 mg/kg/day, intraperitoneal) or an equivalent volume of vehicle was administered to C57 mice for 7 days (Chen et al., 2017), and the mice were subjected to MI/R injury. Compared with the control, it was found that the *in vivo* MI/R injury suppressed AMPK phosphorylation and reduced atrogin-1 levels; however, cardiac CHMP2B levels were elevated. In addition, myocardial LC3 II/I and p62 were accumulated in the MI/R heart, indicating an impaired autophagic flux (Figure 7A). Metformin treatment significantly enhanced AMPK phosphorylation and atrogin-1 levels in the MI/R heart and effectively inhibited CHMP2B accumulation. These effects were associated with decreased LC3 II/I and p62 levels, which indicated the stimulation of autophagic flux (Figure 7A). *In vivo*, metformin treatment enhanced the colocalization of atrogin-1 and CHMP2B in the MI/R heart, as shown by the yellow overlapping area (Figure 7B). Functionally, metformin treatment suppresses cardiac contractile dysfunction (Figures 7C,D), protects the heart from MI/R-induced injury (Figures 7E,F), reduces the arrhythmic severity index (Figure 7G), and significantly decreased the mortality rate in MI/R-injured mice (Figure 7H).

**Figure 7:** Metformin enhancing cardiac AMPK/Atrogin-1 pathways prevent CHMP2B accumulation during MI/R injury. C57 mice were intraperitoneally administered with metformin (100 mg/kg) or vehicle (control) 7 days before MI/R surgery (30 min of ischemia and 2 h of reperfusion). **(A)** Myocardial p-AMPKα, AMPKα, atrogin-1, CHMP2B, p62, and LC3 II/I levels were detected by immunoblots. **(B)** Representative fluorescent images for CHMP2B (green) and atrogin-1 (red) co-localization staining by immunofluorescence in vehicle control or metformin-treated MI/R group. **(C,D)** Representative photomicrographs and average data for left ventricle ejection fraction (LVEF) and fractional shortening (LVFS) were assessed by echocardiography in vehicle control or metformin-treated mice subjected to sham or MI/R injury (30 min of ischemia and 4 weeks of reperfusion). **(E)** LDH concentrations, **(F)** CK-MB activity, and **(G)** arrhythmic index for each group (ischemia 30 min and reperfusion 240 min). **(H)** Survival curve for Con, Ad-CHMP2B, MI/R + Con groups, and MI/R + Ad-CHMP2B groups (*p* ≤ 0.05). Values are means ± SEM, *n* = 6 per group. Except as otherwise noted, *p ≤ 0.05 vs. sham + Ad-Con group. ^#^*p* ≤ 0.05 vs. MI/R + Ad-Con group.

RETRACTED

## Discussion

It is established that CHMP2B plays a crucial role in autophagy. However, the effects of suppressing the elevated CHMP2B levels in the cardiomyocytes during MI/R injury are not known. For instance, when CHMP2B accumulates in the myocardium above the normal threshold, does CHMP2B actually inhibit myocardial autophagy and worsen MI/R injury? Autophagic degradation ability decrease and further accumulation of CHMP2B to form a vicious circle?

We found that excess CHMP2B levels, as seen in CAD patients, resulted in a deficit of myocardial autophagy. This was demonstrated by the elevated LC3 II/I and p62 protein levels during H/R or MI/R injury. Through *in vivo* and *in vitro* experiments, accumulated CHMP2B was shown to induce autophagic flux impairment and, therefore, enhanced myocardial ischemic vulnerability. Here, we demonstrate that CHMP2B is a target of atrogin-1, and atrogin-1 mediates the CHMP2B degradation. Metformin upregulates atrogin-1 levels in MI/R myocardium by activating AMPK, enhancing the interactions between atrogin-1 and CHMP2B, preventing CHMP2B accumulation, improving autophagic flux, and reducing myocardial ischemic injury. In conclusion, CHMP2B is necessary for cardiomyocyte autophagy; however, autophagic disruption can lead to abnormal CHMP2B accumulation. Metformin regulates CHMP2B turnover through the AMPK/atrogin-1 pathways, thereby inhibiting MI/R injury (Supplementary Figure 7).

Myocardial infarction and ischemic heart disease are among the leading global causes of mortality in both the young and elderly population (Virani et al., 2020). The activation of autophagy represents a pro-survival mechanism during myocardial ischemia. Autophagic activation ensures the availability of energy substrates, eliminates damaged mitochondria, and reduces oxidative stress that would otherwise exacerbate myocardial cell death (Shirakabe et al., 2016). Under baseline conditions, autophagy preserves cardiac structure and function. It is activated during stress to limit damage under most conditions. It also reduces injury, preserves cardiac functions during MI/R, inhibits chronic ischemic remodeling, and mediates cardiac adaptation to pressure overload by restricting misfolded protein accumulation. Autophagic impairment is involved in the development of diabetes and aging-induced cardiac abnormalities. We reported on the relationship between autophagic impairment and MI/R injury (Ma et al., 2011; Wang et al., 2019; Li C. et al., 2020). In MI/R-injured myocardium, autophagic impairment leads to p62 accumulation and enhances necroptosis (Li C. et al., 2020). In this study, we confirmed that elevated autophagic signaling protein is attributed to blocked autophagic flux in the MI/R myocardium. This implies a malfunction in protein degradation and turnover during ischemic–reperfusion in the myocardium. Autophagosome clearance is markedly impaired with reperfusion (reoxygenation) in cardiomyocytes after an ischemic (hypoxic) insult, leading to increased abundance of LC3 II/I and p62. This results in an impaired autophagic state that is “ineffective” in cardiac protection against ischemia–reperfusion injury. We found that facilitating autophagic flux by metformin treatment restores functional autophagic processes and attenuates MI/R-induced cardiomyocyte death as well as myocardial dysfunction. The intervention to stimulate a functional autophagic flux confers a protective effect during MI/R.

RETRACTED

The basic mechanism of autophagosome–lysosome fusion in mammalian autophagy has not been fully elucidated. Studies suggest that fusion involves ESCRT (Lee et al., 2009), in which the ESCRT machinery functions in membrane deformation and fission events (Vietri et al., 2020). ESCRT dysfunction has been observed in neurodegeneration (Urwin et al., 2009). Ghazi-Noori et al. (2012) found that transgenic CHMP2B mutant mice had decreased survival rates and exhibited progressive neurodegenerative changes, including gliosis and elevated accumulation of p62- as well as ubiquitin-positive inclusions. These studies have documented that suppressed CHMP2B levels can lead to autophagic dysfunction. However, it is important to determine whether excess CHMP2B inhibits autophagic processes during cardiomyocyte response to stress. We tested this idea and found that CHMP2B is accumulated in H/R *in vitro* and MI/R *in vivo* conditions. Upregulated myocardial CHMP2B, as seen in clinical data of CAD cases, resulted in an autophagic deficit that was demonstrated by the increased LC3-positive puncta fluorescence results with elevated LC3 II/I and p62 protein levels. Functionally, blocking the autophagic flux promoted H/R-evoked cardiomyocyte death *in vitro* and MI/R injury *in vivo*.

RETRACTED

Our study confirmed the harmful effects of excess CHMP2B on the myocardium. Because CHMP2B is necessary for autophagy, CHMP2B knockout is not effective for cardioprotection. Therefore, endogenous degradation of CHMP2B in MI/R myocardium should be promoted. Zaglia et al. (2014) reported that mice lacking atrogin-1 failed to degrade CHMP2B, resulting in autophagic impairment, intracellular protein aggregate accumulation, unfolded protein response activation, and subsequent cardiomyocyte apoptosis, all of which progressively increased with age. However, the upstream regulatory mechanism of myocardial atrogin-1 has not been established. Therefore, can cardioprotection against MI/R injury be ameliorated by regulating atrogin-1-induced CHMP2B degradation?

We found that atrogin-1 and CHMP2B are co-localized in the cardiomyocytes, which was further enhanced by *in vivo* metformin treatment. In addition, the binding relationship between myocardial atrogin-1 and CHMP2B was also shown. CHMP2B is degraded by atrogin-1 through a ubiquitin and time-dependent manner. Abnormalities in CHMP2B degradation contributes to autophagic impairment and cardiac injury. Effectively degrading CHMP2B in the myocardium during MI/R was shown to exhibit cardioprotective effects and reduced mortality in MI/R mice. These results suggest that atrogin-1-dependent degradation of CHMP2B is a novel way of maintaining the homeostasis of autophagic flux. The findings of this study are in concordance with previous reports (Zaglia et al., 2014). CHMP2B aggregates easily, and the gradual accumulation of CHMP2B has the tendency to form amyloid-like complexes that damage cell functions. Metformin treatment is an effective myocardial protective measure that prevents CHMP2B accumulation in MI/R myocardium.

Besides, the relationship between atrogin-1 and CHMP2B in the UPS-autophagy/lysosome system remains elusive. Atrogin-1, also named MAFbx or Fbx32, is a specific muscle-specific E3 ubiquitin ligase in skeletal muscle and myocardium. It is a necessary molecule for mammalian autophagy (Zaglia et al., 2014). CHMP2B is a subunit of ESCRT-III that mediates proteasome degradation and autophagy (Wiersma et al., 2019; Feng et al., 2020). So far as the status, the internal relationship between atrogin-1 and CHMP2B remains elusive. In our article (Figure 5), we clearly prove that CHMP2B is the substrate that is degraded by atrogin-1, and atrogin-1 degrades CHMP2B *via* a ubiquitin-dependent pathway (Figure 5). CHMP2B, as a subunit of ESCRT-III, is a necessary molecule for autophagic homeostasis. In our article, results shown that CHMP2B accumulation impairs cardiac autophagic function and enhances the vulnerability of the cardiac system to ischemia–reperfusion injury. Metformin treatment promotes CHMP2B degradation by atrogin-1 through the AMPK-dependent pathway to maintain the homeostasis of myocardial autophagic flux during MI/R.

RETRACTED

Metformin is a first-line antidiabetic drug that exhibits its cardioprotective effects by promoting autophagy (Li C. et al., 2020). Metformin activates the AMPK pathway and protects against MI/R injury (Wang et al., 2019). In addition, we found that metformin regulates atrogin-1 transcription and expression in an AMPK-dependent manner. Metformin upregulates atrogin-1 in MI/R myocardium by activating AMPK and by enhancing the interaction between atrogin-1 and CHMP2B to degrade CHMP2B and, thereby, protecting autophagy. Metformin treatment also increased cardiac functions and survival rates. Our data extend the previous findings regarding the potential anti-IR effects of metformin. Our registered meta-analysis (CRD42020189905, CRD42020177283, available on PROSPERO) aims to pool clinical evidence for metformin as a therapeutic drug for CVD.

## Study Strengths and Limitations

This study established the harmful effects of CHMP2B accumulation in MI/R injury. Metformin was found to promote CHMP2B degradation through the atrogin-1-dependent pathway. However, some limitations were associated with our study. First, the H9c2 cell line used in this study does not fully conform to the characteristics of primary cardiomyocytes. *In vivo* tissue-derived primary rat cardiomyocytes are better alternatives. Secondly, the transcriptional factor involved in AMPK transcriptional regulation of Atrogin-1 was not determined in our experiments. Previous studies documented that AMPK stimulates atrogin-1 through a forkhead transcription factor in non-primary cardiomyocytes (Nakashima and Yakabe, 2007). More studies should be done to scientifically validate our findings.

## Conclusion

In summary, CHMP2B accumulation impairs cardiac autophagic function and enhances the vulnerability of the cardiac system to ischemia–reperfusion injury. Metformin treatment promotes CHMP2B degradation by atrogin-1 through the AMPK-dependent pathway to maintain the homeostasis of myocardial autophagic flux during MI/R. This is a novel mechanism that enriches the understanding of the mechanisms involved in metformin-AMPK mediated cardioprotection against MI/R injury, especially the regulation of key autophagic factors.

## Data Availability Statement

The original contributions presented in the study are included in the article/Supplementary Materials, further inquiries can be directed to the corresponding author/s.

RETRACTED

## Ethics Statement

Ethical review and approval was not required for the study on human participants in accordance with the local legislation and institutional requirements. Written informed consent for participation was not required for this study in accordance with the national legislation and the institutional requirements. The animal study was reviewed and approved by All animal experiments in this study were approved by the Animal Ethical Experimentation Committee of the Fourth Military Medical University (IACUC-20200602). Written informed consent was not obtained from the individual(s) for the publication of any potentially identifiable images or data included in this article.

## Author Contributions

Conceptualization, investigation, project administration, and supervision: HM, YL, and LY. Data curation: TL and YY. Formal analysis: TL, NM, and YW. Funding acquisition: YY, NM, YW, WJ, LY, and HM. Methodology: ML. Resources: MC. Software: WJ. Validation, visualization, and writing — original draft: TL. Writing — review and editing: HM. All authors contributed to the article and approved the submitted version.

## Conflict of Interest

The authors declare that the research was conducted in the absence of any commercial or financial relationships that could be construed as a potential conflict of interest.
